# Nonlethal age estimation of three threatened fish species using DNA methylation: Australian lungfish, Murray cod and Mary River cod

**DOI:** 10.1111/1755-0998.13440

**Published:** 2021-06-23

**Authors:** Benjamin Mayne, Thomas Espinoza, David Roberts, Gavin L. Butler, Steven Brooks, Darren Korbie, Simon Jarman

**Affiliations:** ^1^ Environomics Future Science Platform Commonwealth Scientific and Industrial Research Organisation (CSIRO) Indian Ocean Marine Research Centre Crawley WA Australia; ^2^ Department of Natural Resources, Mines and Energy Bundaberg Qld Australia; ^3^ Seqwater Ipswich Qld Australia; ^4^ Department of Primary Industries Grafton Fisheries Centre Grafton NSW Australia; ^5^ Department of Agriculture, Fisheries and Forestry Brisbane Qld Australia; ^6^ Australian Institute for Bioengineering and Nanotechnology The University of Queensland Brisbane Qld Australia; ^7^ School of Biological Sciences The University of Western Australia, Crawley WA Australia

**Keywords:** age estimation, DNA methylation, epigenetic Clock, fish, wildlife management

## Abstract

Age‐based demography is fundamental to management of wild fish populations. Age estimates for individuals can determine rates of change in key life‐history parameters such as length, maturity, mortality and fecundity. These age‐based characteristics are critical for population viability analysis in endangered species and for developing sustainable harvest strategies. For teleost fish, age has traditionally been determined by counting increments formed in calcified structures such as otoliths. However, the collection of otoliths is lethal and therefore undesirable for threatened species. At a molecular level, age can be predicted by measuring DNA methylation. Here, we use previously identified age‐associated sites of DNA methylation in zebrafish (*Danio rerio*) to develop two epigenetic clocks for three threatened freshwater fish species. One epigenetic clock was developed for the Australian lungfish (*Neoceratodus forsteri*) and the second for the Murray cod (*Maccullochella* *peelii*) and Mary River cod (*Maccullochella* *mariensis*). Age estimation models were calibrated using either known‐age individuals, ages derived from otoliths or bomb radiocarbon dating of scales. We demonstrate a high Pearson's correlation between the chronological and predicted age in both the Lungfish clock (cor = .98) and *Maccullochella* clock (cor = .92). The median absolute error rate for both epigenetic clocks was also low (Lungfish = 0.86 years; *Maccullochella* = 0.34 years). This study demonstrates the transferability of DNA methylation sites for age prediction between highly phylogenetically divergent fish species. Given the method is nonlethal and suited to automation, age prediction by DNA methylation has the potential to improve fisheries and other wildlife management settings.

## 1 INTRODUCTION

Information on the age structure of fish populations is valuable for making accurate predictions of future population growth rates (Berkeley et al., 2004; Caughley, 1977a; Udevitz & Ballachey, 1998). Age is fundamental to determine key life‐history parameters such as age‐at‐length, age of reproductive maturity, age‐related mortality and fecundity (Das, 1994; Žák & Reichard, 2021). The age of teleost fish has traditionally been estimated by counting growth increments (rings) in hard structures such as otoliths, vertebrae, fin spines and scales. Otoliths (ear bones) are the most common structure used and are considered more accurate than other metabolically active structures (Campana & Thorrold, 2001). However, not all teleost fish species exhibit otolith growth increments or other phenotypic age characteristics, making it more difficult to monitor the population dynamics for those species (Gauldie et al., 1986; Iizuka & Katayama, 2008). The extraction of otoliths for age estimation is also a lethal process, making it undesirable for application to threatened or endangered species. Another limitation of otoliths is the difficulty in ageing both the youngest and the oldest fish (Campana, 2001). The difficulty in ageing an otolith can also introduce reader bias, potentially having an impact on any population management (Campana, 2001). Where otoliths or other ageing methods are not applicable; an alternative nonlethal approach to age estimation is required to better manage wild populations.

The iconic and phylogenetically significant Australian lungfish (*Neoceratodus forsteri*) is an example of a threatened species whose age cannot be reliably estimated using otoliths (Gauldie et al., 1986). Australian lungfish are often referred to as living fossils and belong to a group that evolved at least 380 million years ago, at a time when vertebrate classes were diversifying (Bailes et al., 2007; Brinkmann et al., 2004). Their unique evolutionary position, restricted natural distribution and conservation status warrant efforts to develop a reliable nondestructive age determination method to aid in conservation (Espinoza et al., 2019). Bomb radiocarbon techniques have been used previously to estimate age in Australian lungfish (Fallon et al., 2019). Although bomb radiocarbon is an effective method to determine age, it can be expensive thus making it difficult to routinely estimate age in large populations. This method is expensive and may also be affected by environmental parameters, such as carbon isotope composition of the food or environment, that may confound interpretation and calibration in some fish species.

Ageing via otoliths has been the most reliable and common method utilized to date for many threatened freshwater fish, including the vulnerable Murray cod (*Maccullochella peelii*) and endangered Mary River cod (*Maccullochella mariensis*) (Couch et al., 2016; Espinoza et al., 2019). These two species are endemic to the Murray and Mary river systems of eastern Australia. They are large apex predators and have important cultural significance to indigenous and nonindigenous Australians. However, both species have declined significantly in range and abundance as a result of overfishing and water regulation (Koehn, 2004; Lintermans et al., 2005; Stewardson & Skinner, 2018). Using otoliths to age threatened species could be considered inconsistent with conservation goals and can impose practical limits on sample sizes and thus representativeness of age estimates for a population (Smart et al., 2013).

In mammals, birds and fish, epigenetic methods have been used to determine age (Anastasiadi & Piferrer, 2020; De Paoli‐Iseppi et al., 2019; Horvath, 2013; Mayne et al., 2020; Polanowski et al., 2014; Stubbs et al., 2017; Thompson et al., 2017; Wright et al., 2018). The most common form of DNA methylation in vertebrates is the addition of a methyl group to cytosines within cytosine‐phosphate‐guanine (CpG) sites (Bird, 1993). DNA methylation for age estimation is measured in blood, saliva or skin as this offers a nonlethal approach (De Paoli‐Iseppi et al., 2017). Historically, a limitation of using DNA methylation to estimate age in animals was the high cost of characterizing large fractions of the genome. However, short read sequencing has reduced costs significantly in recent years (Heather & Chain, 2016; Li et al., 2019).

The *de novo* identification of informative methylation markers for a new species typically involves a significant investment in DNA sequencing on known‐age specimens (Mayne et al., 2020; Stubbs et al., 2017; Thompson et al., 2017). This results in many candidate markers that are informative for age, though typically a much smaller fraction is required to reliably age specimens. Previous studies have used three to 353 CpG sites for their epigenetic clocks (Horvath, 2013; Polanowski et al., 2014). The total number of CpG sites needed for epigenetic clocks is dependent upon many factors, including but not limited to, single or multitissue type, assay design (microarray vs. sequencing), biological variability and technical variability. An alternative, and more cost‐effective approach to development of markers is to transfer them among taxa. In humpback whales (*Megaptera novaeangliae*) and Bechstein's bats (*Myotis bechsteinii*), age estimation models were developed using conserved age‐associated CpG sites in humans and mice (*Mus musculus*) (Polanowski et al., 2014; Wright et al., 2018). In a recent study, it has been found that CpG sites across 128 mammalian species can be predictive of age (Mammalian Methylation Consortium et al., 2021). This study highlights the potential to generate universal epigenetic clocks and the evolutionary conservation of CpG sites with ageing across a broad range of species. The maintenance of age‐association in conserved CpG sites between relatively distantly related mammalian species suggests an underlying common mechanistic basis. The transfer of age‐informative CpG markers has not been tested in other vertebrate groups, and specifically in groups such as bony fishes (Osteichthyes) that possess significantly greater phylogenetic depth than eutherian mammals. In the present study, we use age‐associated CpG sites identified in zebrafish (*Danio rerio*) to develop two age estimation models for three threatened fish species. The first epigenetic clock presented in this study is for the Australian lungfish and the second for the Murray cod and Mary River cod. Fin tissue was used to develop the model for each species, thereby making the method nonlethal. The approach provides an alternative to bomb radiocarbon and otolith ageing and is well suited to use on threatened and exploited species.

## 2 MATERIALS AND METHODS

### 2.1 Animal ethics and tissue collection

Australian lungfish samples were collected from the Brisbane, Burnett and Mary rivers in southeast Queensland, Australia. Collection of fin tissue was approved under General Fisheries Permits 174232 and 140615 and approved by Australian Ethics Committee protocol numbers CA2011/10/551 and ENV/17/14/AEC. A mix of Australian lungfish samples of known age and age determined by bomb radiocarbon dating were used in this study (Table 1) (Fallon et al., 2015; James et al., 2010). The known‐age Australian lungfish samples were used from previous research projects and mortalities of captive‐raised and Convention on International Trade in Endangered Species (CITES)‐registered fish including public aquarium and private aquarium collections (Fallon et al., 2019).

**TABLE 1:** Total number of samples and age ranges used for Australian lungfish (*Neoceratodus forsteri*), Mary River cod (*Maccullochella mariensis*) and Murray Cod (*Maccullochella peelii*)

Species	Total samples	Age range (years)
Australian lungfish (*Neoceratodus forsteri*)	141 (102 bomb radiocarbon age and 39 known age)	bomb radiocarbon age: 2–77 known age: 0.1–14
Mary River cod (*Maccullochella mariensis*)	37 (37 known age)	0.5–2.88
Murray cod (*Maccullochella peelii*)	33 (33 otolith age)	1.1–12.1

Collection of fin tissue from known‐age Mary River cod was approved under General Fisheries Permit 94765 and Animal Ethics Permit CA 2008/03/253 from wild and captive raised fish. Murray cod otoliths and fin tissue were collected from multiple rivers along the Queensland and New South Wales border within the Border Rivers region of the Northern Murray–Darling Basin. Collection of fin tissue was approved by CA 2019/04/1276 and otoliths under NSW Animal Research Authority 10/04. Otolith ageing of Murray cod was conducted using a previous validated method (Gooley, 1992). Table 1 lists the total number and age ranges used for both Murray cod and Mary River cod.

### 2.2 DNA extraction and bisulphite treatment

DNA was extracted using the DNeasy Blood & Tissue Kit (Qiagen) according to the manufacturer's protocol. DNA quality was assessed using the 260/280 ratio with ratios of ~1.8 considered being pure DNA (Qiaxpert; Qiagen). Bisulphite treatment was performed as described previously with 150 ng of extracted DNA (Clark et al., 2006).

### 2.3 Primer design

For both models, primers were designed by targeting CpG sites with methylation levels that are both known to significantly correlate with age in zebrafish and conserved between zebrafish and our target species. Previously, 1,311 CpG sites were found to have methylation levels that significantly correlate with age in zebrafish (Pearson correlation, *p* < .05, Table S1) (Mayne et al., 2020). These sites were identified as being age‐associated by generating a reduced representation bisulphite sequencing (RRBS) data set of caudal fin tissue from known‐age zebrafish. In this study, we develop specific epigenetic clocks for the Australian lungfish and the Mary River cod and Murray cod as opposed to a universal clock, demonstrated in mammals (Mammalian Methylation Consortium et al., 2021). The rationale for this is that we were unable to identify conserved age‐associated CpG sites across the three fish species through genome pairwise alignments. There was no conservation of CpG sites in the two epigenetic clocks presented in this study. The conservation of CpG sites was only between zebrafish and the species of interest.

At the time this study was conducted a reference genome for the Australian lungfish was unavailable. We therefore used publicly available RNA‐sequencing (RNA‐seq) data (BioProject accession ID: PRJNA282925) as a substitute for genomic data (Biscotti et al., 2016). hisat2 version 2.1.0 with default parameters was used to align the RNA‐seq data to the zebrafish reference genome (danRer10, Illumina iGenomes) (Kim et al., 2015). RNA‐seq alignments that overlapped with age‐associated CpG sites identified by bedtools version 2.25.0 were targeted for primer design (Table S2).

The Mary River cod and Murray cod have a median divergence time of 1.09 million years ago (Ma) (Nock et al., 2010). Due to the low evolutionary divergence time between the species and the Murray cod being the only one with a reference genome, the primers were designed using the Murray cod genome (GCA002120245.1 mcod version 1, https://www.ncbi.nlm.nih.gov/genome/24609) but were also used on the Mary River cod (Austin et al., 2017). CpG sites conserved between the zebrafish and Murray cod genomes were identified with lastz version 1.04.00 with the following conditions: [multiple]–notransition–step = 20–nogapped (Harris, 2007). Conserved DNA sequences between the two genomes with methylation age‐associated CpG sites were targeted for primer design (Table S3).

### 2.4 Singleplex and multiplex PCR

Primer pairs were designed using primersuite and for one PCR pool (Lu et al., 2017). The ligating sequence for the primers is represented as lower‐case bases in Tables S2 and S3. Primers were tested individually using the GoTaq Hot Start Polymerase (Promega) as recommended in the manufacturer's cycling conditions. Primer pairs that produced one product at the predicted size were used together as a multiplex PCR (Australian lungfish: 13 primer pairs successful; Murray and Mary River cod: 26 primer pairs successful). The final multiplex PCR details are provided in Table S4. The multiplex PCR cycling conditions were: 94°C, 5 min; 12 cycles (94°C, 20 s; 60°C, 60 s); 16 cycles (94°C, 20 s; 65°C, 90 s); 65°C, 3 min; 4°C hold. Gel electrophoresis with sodium borate buffer using a 1.5% agarose gel was used to visualize PCR products.

### 2.5 Barcoding and sequencing

Barcoding of samples occurred with oligonucleotides with attached MiSeq adaptors (Fluidigm, 100–4876). The reaction details are provided in Table S5. The cycling conditions for barcoding were: 94°C, 5 min; 12 cycles (97°C, 15 s; 45°C, 30 s; 72°C 2 min); 72°C, 2 min; 4°C hold. Barcoding was performed using an Eppendorf ProS 96. The Illumina MiSeq Reagent Kit version 2 (300 cycles; PN MS‐102–2002) was used for 150‐bp paired‐end sequencing.

### 2.6 Data analysis and age estimation

seqkit version 1.2 was used to hard clip the reads by 15 bp at both 5′ and 3′ ends to remove adaptor sequences (Shen et al., 2016). Reads were aligned to a reduced representation of a genome of each species’ closest relative. Here the genome was partitioned into only sequences that contained the age‐associated CpG sites, thereby reducing computational time. Lungfish reads were aligned to the zebrafish genome. The sequencing captured 31 CpG sites in the Australian lungfish. Both the Murray cod and Mary River cod were aligned to the Murray cod genome (GCA002120245.1 mcod version 1) and captured 26 CpG sites. bismark version 0.20.0 was used to align reads with the following parameters: ‐‐bowtie2‐N1‐L15–bam‐p2–score L, −0.6, −0.6 –non_directional. Methylation calling was performed using the bismark_methylation_extractor function with default parameters (Krueger & Andrews, 2011).

For each model, 70% of the samples were randomly assigned to a training data set and the remainder into a testing data set similar to the approach of previous studies (Horvath, 2013; Mayne et al., 2020; Stubbs et al., 2017; Thompson et al., 2017). The advantage of the 70/30 split is that it sets aside data to test for overfitting. This is ideal in models that may have future application. Age in years was natural log‐transformed and an elastic net regression model was applied to the training data sets. Age was regressed over the methylation of each CpG site that was captured during sequencing. The glmnet function used for the elastic net regression model was set to a 10‐fold cross‐validation with an α‐parameter = 0 (Friedman et al., 2010). The α‐parameter was set to 0 as this forces all sites to be used in the model, as opposed to other studies where it is set to 0.5 to identify the minimum number of sites required (Horvath, 2013; Mayne et al., 2020; Stubbs et al., 2017; Thompson et al., 2017). This is because in this study, unlike previous studies that have captured thousands of CpG sites, we only had a limited number available (Horvath, 2013; Mayne et al., 2020; Stubbs et al., 2017; Thompson et al., 2017). Ideally, assessing a higher number of CpG sites may capture better predictors of age. However, in this study we aimed to transfer known‐age associated CpG sites between species to prevent the need to perform expensive genome‐wide sequencing. A one‐way analysis of variance (ANOVA) was used to test if the absolute error rate was higher with samples from known‐age or bomb radiocarbon age. All analyses were performed in R version 3.5.1 (Team, 2006).

## 3 RESULTS

### 3.1 Generating age estimation models

In total, 11.1 million reads were generated for the 211 sequenced samples. An average of 41,635 reads per sample were aligned to the respective reference genome with an average alignment rate of 97.5%. For the Australian lungfish, 31 CpG sites were used to calibrate the age estimator model and will be referred to as the Lungfish clock (Table S6). For the Murray and Mary River cod 26 CpG sites were used to calibrate the model and will be referred to as the *Maccullochella* clock (Table S7).

### 3.2 Lungfish clock

For the Lungfish clock we found a high correlation between the chronological age and the predicted age in both the training (Pearson correlation = .98, *p* < 2.20 × 10^−16^) and the testing data set (Pearson correlation = .98, *p* < 2.20 × 10^−16^; Figure 1a,b). The median absolute error (MAE) in the testing data set was 0.86 years (Figure 1c). No significant difference in MAE was found between the training and testing data sets (*p* = .67, *t* test, two‐tailed). The similar correlation in chronological and predicted age and no significant difference in MAE suggests a lack of overfitting in the model. A higher performance of the model was observed at younger ages (Table 2). The Pearson correlation between the chronological and predicted age decreased and the MAE and relative error increased with age. We also tested if the epigenetic clock performed better with samples of known age or bomb radiocarbon age. Chronological age was used as a blocking factor as most younger ages were of known age (Table 1). We found no significant difference between the error rate of samples from known or bomb radiocarbon age for both the training (*p* = .413, one‐way ANOVA) and the testing data set (*p* = .803).

**FIGURE 1:** Age estimation by DNA methylation in the Australian Lungfish. Correlation plots between the chronological and predicted age in the (a) training data set (Pearson correlation = 0.98, *p*‐value < 2.20 × 10^−16^) and (b) testing data set (Pearson correlation = 0.98, *p*‐value < 2.20 × 10^−16^). (c) Boxplots show the absolute error rate in age estimation in both the training and testing data sets

**TABLE 2:** Performance of the Lungfish and *Maccullochella* epigenetic clocks at increasing age intervals in the testing data set

Age range	Correlation	Median absolute error (years)	Median relative error (%)
Lungfish clock			
≤20	.99	0.16	8.44
21–40	.85	2.65	7.82
41–60	.71	6.90	12.52
>60	.60	6.09	9.30
*Maccullochella* clock			
≤5	.98	0.35	9.16
6–10	.25	1.99	28.10
>10	.08	2.86	24.04

Note

The absolute and relative error rates for each age range is reported as the average (median). Relative error was calculated by dividing the absolute error by the chronological age and is expressed as a percentage.

### 3.3 *Maccullochella* clock

We found a high correlation between the chronological and predicted age in both the training (Pearson correlation = .92, *p* < 2.20 × 10^−16^) and the testing data set (Pearson correlation = .92, *p*‐value = 5.97 × 10^−13^) (Figure 2a,b). A low MAE of 0.34 years was observed in the testing data with no significant difference in the training data set (*p* = .53, *t* test, two‐tailed; Figure 2c). As described for the lungfish, the similar correlation values and low MAE in the training and testing data sets suggests a lack of overfitting by the model.

**FIGURE 2:** Age estimation by DNA methylation in the Murray cod and Mary River cod. Correlation plots between the chronological and predicted age in the (a) training data set (Pearson correlation < 0.92, *p*‐value < 2.20 × 10^−16^) and (b) testing data set (Pearson correlation = 0.92, *p*‐value = 5.97 × 10^−13^). (c) Boxplots show the absolute error rate

To test if the model was performing better on either the Murray cod or Mary River cod, a one‐way ANOVA was used with chronological age as a blocking factor. A blocking factor was used to reduce bias between the age of samples as all samples above 2.9 years were Murray cod. No difference was found between the species in both the training (*p* = .139, one‐way ANOVA) and the testing data set (*p* = .185). This suggests the model performance is not biased towards one species. Likewise, as in the Lungfish clock, we found the performance of the *Maccullochella* clock to be highest with younger individuals (Table 2).

## 4 DISCUSSION

We have developed two epigenetic clocks for three threatened fish species. These epigenetic clocks can be applied nonlethally using fin clips taken from fish. Our approach transferred age‐associated CpG sites characterized previously in a model species, the zebrafish, to deeply phylogenetically divergent fish taxa (Mayne et al., 2020). Despite an evolutionary divergent time of up to 433 Ma, we demonstrate highly accurate and precise epigenetic clocks for our target species (Kumar et al., 2017).

The use of epigenetic clocks in wildlife management has many advantages. First, epigenetic clocks are relatively inexpensive when analysing large sample numbers, compared to techniques such as bomb radiocarbon. In terms of sequencing alone, when running with 384 samples per Illumina MiSeq run the cost was approximately $5 (AUD) in reagent costs. Second, epigenetic clocks are nonlethal, unlike otolith reading. Third, epigenetic clocks are not hindered by a manual reader or rely on differentiating ever declining concentrations of atmospheric radiocarbon. In otolith age estimation, a reader bias may be difficult to estimate but even small errors may have an impact on the overall management of a population (Campana, 2001; Moen et al., 2018). The determination of catch and size limits in fisheries management is dependent upon nonbiased age structure (Brunel & Piet, 2013). It is therefore critical to have an accurate and precise method for age determination. By being both inexpensive and nonlethal, epigenetic clocks have potential to be of significant value in the field of fisheries management. For example, in threatened species it may be impossible to determine an age structure of a population. Without an age structure, the population growth, risk of extinction and other population dynamics cannot be accurately defined (Caughley, 1977b).

As was found in this study, epigenetic clocks that have been calibrated on one species have been shown to predict age accurately in closely related species. For example, the human epigenetic clock transferred to chimpanzees (*Pan troglodytes*), with a median evolutionary distance of 6.4 Ma (Horvath, 2013; Kumar et al., 2017). The advantage of developing the *Maccullochella* clock with two species is the potential use of age estimation for other members of the genus *Maccullochella*. The time separating the last common ancestor for the *Maccullochella* genus ranges between 4.35 and 9.99 Ma (Nock et al., 2010). The genus *Maccullochella* comprises four species: Murray cod, Mary River cod, eastern freshwater cod (*Maccullochella ikei*) and trout cod (*Maccullochella macquariensis*) (Nock et al., 2010). The *Maccullochella* clock has the potential to be used to estimate the ages of eastern freshwater cod and the trout cod despite the model not being calibrated with either species. However, whilst it is most probably applicable to these other two species and potentially others, we recommend that samples with known ages should be tested prior to using the *Maccullochella* clock for any other species applications.

One of the challenges to using DNA methylation as a predictive measure of age is the necessity of training the model using a large data set. The Australian lungfish data set consisted of 102 bomb radiocarbon samples and 39 known‐age samples up to 77 years of age. Therefore, a degree of caution should be taken with using the model on long‐lived lungfish as the model was only trained with ages up to 77 years. A similar approach should be taken for the *Maccullochella* clock. The *Maccullochella* clock was trained with a mix of known and estimated ages up to 12.1 years, but Murray cod have been reported as old as 48 years (Anderson et al., 1992). One of the challenges with using DNA methylation as a predictor of age is the decrease in accuracy with higher ages. As shown in Table 2, the performance of both models decreases with increasing age. The model could potentially be improved in future research when older known‐age individuals become available. Better prediction of age among younger individuals has been observed in previous epigenetic clocks (Shireby et al., 2020). Biological ageing may influence epigenetic clocks at older ages, lowering the predictive power for chronological age of the model (Bell et al., 2019). Another option would be to log‐transform only younger individuals in the model calibration, similar to an approach used previously with the human epigenetic clock (Horvath, 2013). This can improve the performance of age estimation in older individuals. In the specific case of this study, determining a cut‐off to log‐transform the young ages is not simple as the age gap increases with age. This may result in an over correction or bias in the model. However, for a data set with a uniform distribution of ages, log‐transformation of younger ages may improve the accuracy of estimates. Ideally, both models would benefit from a larger sample size of known‐age fish. However, many ecological studies have to work with what is available and the data sets used in this study are the largest epigenetic clocks developed to date in wild animals (Anastasiadi & Piferrer, 2020; De Paoli‐Iseppi et al., 2017). DNA methylation ageing provides additional opportunities for ongoing age verification of species with limited population size, through mark–recapture and tissue sampling to expand the age range of the model, and to verify known ages as the marked fish age. This is not possible with destructive ageing techniques.

One of the major challenges in developing epigenetic clocks is the choice of CpG sites. Studies take either a genome‐wide approach or a targeted approach for CpG selection. This study has taken sites from a previous genome‐wide study in zebrafish and then used evolutionary conserved sites between species (Mayne et al., 2020). An epigenetic clock in European seabass (*Dicentrarchus labrax*) used a targeted approach for CpG site selection (Anastasiadi & Piferrer, 2020). Although multiple methods to develop epigenetic clocks for fish have been demonstrated here and, in the literature, this study shows the potential to transfer sites between distantly related species. The rapid transfer of age‐associated sites to develop new epigenetic clocks has the potential to improve the wildlife management for a broader range of fish species.

We demonstrate here the utility of epigenetic clocks to nonlethally and accurately predict age in closely and divergent related fish species. Epigenetic clocks can provide a new and significantly improved method for characterizing the age structure of potentially numerous commercial, recreational and conservation significant species. This demonstration of using age‐associated sites between species that are separated by up to 433 million years provides confidence that the methodology can be applied across a broad range of fish species. Epigenetic clocks have the potential to greatly advance fisheries management and allow the ageing of species formerly sensitive for large‐scale lethal sampling to provide representative population age structures.

## CONFLICT OF INTEREST

The authors have no conflicts of interest to declare.

## AUTHOR CONTRIBUTIONS

BM performed all laboratory work, bioinformatic analysis, performed the machine learning analysis to generate each age estimation model and wrote the manuscript. TM, DR, GB, and SB collected the fin clips from the fish used in the study and provided discussion, intellectual input into the manuscript. DK designed the primers for the multiplex PCR and was involved in the study design. SJ was involved in the study design, provided discussion, and intellectual input into the manuscript. All authors read and approved the final version of the manuscript.

## Supporting information

Table S1‐S3

Supplementary Material

## Data Availability

Multiplex PCR followed by sequencing data are publicly available at https://data.csiro.au/collections/collection/CIcsiro:49713v1
